# 3′,4′-Dihydroxyflavonol Antioxidant Attenuates Diastolic Dysfunction and Cardiac Remodeling in Streptozotocin-Induced Diabetic m(Ren2)27 Rats

**DOI:** 10.1371/journal.pone.0022777

**Published:** 2011-07-28

**Authors:** Fay Lin Khong, Yuan Zhang, Amanda J. Edgley, Weier Qi, Kim A. Connelly, Owen L. Woodman, Henry Krum, Darren J. Kelly

**Affiliations:** 1 Department of Medicine, The University of Melbourne, St Vincent's Hospital Fitzroy, Melbourne, Victoria, Australia; 2 St Vincent's Institute of Medical Research, St Vincent's Hospital Fitzroy, Melbourne, Victoria, Australia; 3 School of Medical Sciences, Royal Melbourne Institute of Technology (RMIT) University Bundoora, Melbourne, Victoria, Australia; 4 Department of Medicine, St Michael's Hospital, Toronto, Ontario, Canada; 5 Department of Epidemiology and Preventive Medicine and Department of Medicine, Faculty of Medicine, Nursing and Health Sciences, Centre of Cardiovascular Research & Education (CCRE) in Therapeutics, Monash University, The Alfred, Melbourne, Victoria, Australia; Pennington Biomedical Research Center, United States of America

## Abstract

**Background:**

Diabetic cardiomyopathy (DCM) is an increasingly recognized cause of chronic heart failure amongst diabetic patients. Both increased reactive oxygen species (ROS) generation and impaired ROS scavenging have been implicated in the pathogenesis of hyperglycemia-induced left ventricular dysfunction, cardiac fibrosis, apoptosis and hypertrophy. We hypothesized that 3′,4′-dihydroxyflavonol (DiOHF), a small highly lipid soluble synthetic flavonol, may prevent DCM by scavenging ROS, thus preventing ROS-induced cardiac damage.

**Methodology/Principal Findings:**

Six week old homozygous Ren-2 rats were randomized to receive either streptozotocin or citrate buffer, then further randomized to receive either DiOHF (1 mg/kg/day) by oral gavage or vehicle for six weeks. Cardiac function was assessed via echocardiography and left ventricular cardiac catheterization before the animals were sacrificed and hearts removed for histological and molecular analyses. Diabetic Ren-2 rats showed evidence of diastolic dysfunction with prolonged deceleration time, reduced E/A ratio, and increased slope of end-diastolic pressure volume relationship (EDPVR) in association with marked interstitial fibrosis and oxidative stress (all *P*<0.05 vs control Ren-2). Treatment with DiOHF prevented the development of diastolic dysfunction and was associated with reduced oxidative stress and interstitial fibrosis (all *P*<0.05 vs untreated diabetic Ren-2 rats). In contrast, few changes were seen in non-diabetic treated animals compared to untreated counterparts.

**Conclusions:**

Inhibition of ROS production and action by DiOHF improved diastolic function and reduced myocyte hypertrophy as well as collagen deposition. These findings suggest the potential clinical utility of antioxidative compounds such as flavonols in the prevention of diabetes-associated cardiac dysfunction.

## Introduction

The association between diabetes and cardiovascular disease is beyond dispute, with diabetes being an independent risk factor for the development of cardiovascular complications, accounting for 80% of deaths among diabetic patients [1], [2], [3]. However the mechanisms underlying the development of chronic heart failure (CHF) in diabetic patients remain uncertain. A large body of evidence demonstrates that diabetic cardiomyopathy (DCM) exists, independent of hypertension and underlying coronary artery disease [4], [5]. DCM is characterized particularly by fibrosis and hypertrophy in the left ventricle (LV) of the heart manifested as abnormal LV diastolic function preceding LV systolic dysfunction [3], [6], [7].

While the mechanisms underlying these pathological changes are not well understood, reactive oxygen species (ROS) have been identified as likely mediators in the pathophysiology of diabetic cardiovascular complications [8]. During the progression of DCM, depletion of endogenous antioxidant reserves and hyperglycemia-induced ROS generation causes a state of oxidative stress [9]. Hyperglycemia-induced overproduction of superoxide by the mitochondrial electron-transport chain seems crucial to the activation of various metabolic pathways implicated in diabetic subjects. Superoxide overproduction is accompanied by increased nitric oxide generation favouring the formation of the reactive oxidant peroxynitrite which induces damage to biomacromolecules i.e. lipid peroxidation and protein oxidation and nitration [10], [11]. Also, activation of ROS-generating NADPH oxidase isoforms in the heart by various stimuli during hyperglycemia including angiotensin II (Ang II), endothelin-1 (ET-1), cytokines and growth factors, appears to be important in redox-sensitive signalling leading to the accumulation of extracellular matrix (ECM) proteins, interstitial and perivascular fibrosis and myocyte hypertrophy causing LV remodelling [12], [13], [14], [15].

Current evidence-based therapies for the treatment of diabetes and cardiac disease, including ACE inhibitors, angiotensin receptor blockers (ARB), and statins have some intracellular antioxidant activity [16]. Despite the abovementioned treatments and intensive glucose or blood pressure control, CHF remains a major public health burden with the need for new therapeutic strategies. Flavonols are plant-derived polyphenolic compounds that have been recognized to not only scavenge intracellular and extracellular ROS but to also inhibit enzymes responsible for the production of superoxide anions including xanthine oxidase, NADPH oxidase, cyclooxygenase, lipoxygenase, and protein kinase C [17], [18]. Recently, DiOHF (3′,4′-dihydroxyflavonol), a small highly lipid soluble synthetic flavonol, has been demonstrated to attenuate myocardial ischemia/reperfusion injury, associated with its antioxidant activity [19], [20]. However, the antioxidant actions of orally administered DiOHF have yet to be tested in the setting of hyperglycemia-induced DCM.

Accordingly, the present study aimed to examine the effects of DiOHF on cardiac function and structure in experimental DCM. The study was undertaken in the streptozotocin-induced transgenic m(Ren-2)27 rat, a hemodynamically validated model of diabetes-induced diastolic heart failure, which has been shown to develop structural and functional changes similar to that observed in human DCM [21], [22]. We demonstrated that DiOHF effectively reduced cardiac oxidative stress and was cardioprotective against cardiac dysfunction that develops as a consequence of diabetes.

## Materials and Methods

### Ethics statement

Experimental procedures were approved by the St Vincent's Hospital Animal Ethics Committee, Melbourne, Australia in accordance with the National Health and Medical Research Council of Australia's Code of the Care and Use of Animals for scientific purposes: Ethics Approval ID. 063/03 (PC2 certificate number. 1480/2003, Permit number. SPPL120).

### Animals and procedures

Six week old male homozygous transgenic m(Ren-2)27 rats (St. Vincent's Hospital Animal Resource Centre, Melbourne, Victoria, Australia) were randomized to receive either 55 mg/kg of streptozotocin (STZ; Sigma, St Louis, MO, USA) diluted in 0.1 mol/L citrate buffer pH 4.5 (diabetic) to induce experimental type 1 diabetes or citrate buffer alone (non-diabetic control) by tail vein injection following overnight fasting. Diabetic and control rats (n = 10) were further randomized to receive either an orally active synthetic antioxidant, DiOHF (3′,4′-dihydroxyflavonol; Indofine Chemical Co., USA) at 1 mg/kg or vehicle (1% carboxy methyl cellulose solution; CMC) by daily gavage for six weeks post STZ. DiOHF was a gift from NeuProtect Pty Ltd, Melbourne VIC. Animals were housed in a stable environment maintained at 21±1°C (12 hour light/dark cycle commencing at 6 am). Animals had free access to standard rat chow (GR2 Clark-King and Co, Gladesville, NSW, Australia) and drinking water.

Each week, rats were weighed and their blood glucose levels were measured (Accucheck Advantage II Blood Glucose Monitor, Roche Diagnostics, USA). Only STZ-treated animals with blood glucose greater than 15 mmol/L were considered diabetic. Prior to the induction of diabetes and every three weeks post randomization, systolic blood pressure (SBP) was assessed in preheated conscious rats by tail cuff plethysmography using a non-invasive blood pressure controller and Powerlab system (AD Instruments Pty Ltd, NSW, Australia) [23], [24]. Diabetic animals received 2–4 units of isophane insulin (Humulin NPH; Eli Lilly and Co., NSW, Australia) intraperitoneally 3 times per week to maintain blood glucose levels, promote weight gain and reduce mortality.

At the end of the experimental period, animals were anaesthetized (pentobarbitone sodium 30 mg/kg body weight i.p.; Virbac, Peakhurst, NSW, Australia). The abdomen, neck, and chest were shaved, and echocardiography performed followed by in vivo left ventricular pressure-volume loop acquisition.

### Echocardiography

Detailed two dimensional and Doppler echocardiography were performed to assess systolic and diastolic function using a Vivid 7 Dimension (GE Vingmed, Horten, Norway) echocardiograph with a 10 MHz phased array probe, as previously published [21]. Animals underwent echocardiographic interrogation in the left recumbent position, after being anaesthetized using the protocol above. All data were acquired and analyzed by a single blinded observer using EchoPAC (GE Vingmed) offline processing.

### Cardiac catheterization

Cardiac catheterization was performed as previously published [21]. Post echocardiography, animals were placed on a warming pad (37°C), intubated using a 14 gauge catheter, and ventilated using positive pressure with a tidal volume of 8 to 10% body weight at 70 breaths/min using room air. The right internal carotid artery was identified, ligated, and a 2F miniaturized combined conductance catheter-micromanometer (Model SPR-838 Millar instruments, Houston, TX) was inserted to obtain aortic blood pressure, then advanced into the LV until stable PV loops were obtained. Data were acquired under steady state conditions and during preload reduction. Using the pressure conductance data, a range of functional parameters was then calculated (Millar analysis software PVAN 3.4). These included end diastolic pressure (EDP), end systolic pressure (ESP), the time constant of the isovolumic-pressure decline (Tau, τ Weiss), the slope of end diastolic pressure volume relationship (EDPVR), and the slope of the preload recruitable stroke work relationship (PRSW), defined as the relationship between stroke work (SW) and end diastolic volume (EDV) [21]. The active and passive phases of diastole were resolved by the assessment of Tau and EDPVR, respectively.

### Tissue collection

Animals were euthanized with a further dose of anaesthetic (pentobarbitone sodium 60 mg/kg of body weight i.p.; Virbac, Peakhurst, NSW, Australia) and their hearts and lungs excised. The whole heart and lung were blotted dry and weighed. The heart was then dissected into atria, right ventricle and left ventricle, inclusive of the interventricular septum, and weighed separately. The apex was removed, bisected and snap frozen in −80°C liquid nitrogen for chemiluminescence. The top portion of the LV was fixed in 10% neutral buffered formalin overnight for subsequent processing and the mid portion was embedded in Tissue-Tek® OCT compound (Sakura Finetek USA, Inc., Torrance, CA, USA) and stored in a −80°C freezer. The formalin-fixed LV sections were paraffin-embedded and sectioned to 4 µm thick using a rotary microtome (Leica Microsystems GmbH Wetzlar, Germany).

### Histopathology and immunohistochemistry

Changes in cardiac structure were assessed in a masked protocol in at least 10 randomly selected tissue sections from each group studied. Sections were stained with picrosirius red to demonstrate collagenous matrix and fibrillar collagen types I and III were assessed using specific antibodies (anti-type I collagen 1∶100: Southern Biotechnology Associates Inc., Birmingham, AL, USA; anti-type III collagen antibody: Biogenex, San Ramon, CA, USA). Indication of oxidative damage within the myocardium was assessed using anti-nitrotyrosine 1∶40 (Upstate, NY, USA). In brief, 4 µm LV sections were dewaxed in histolene, rehydrated in graded ethanol, and immersed in distilled water. Each LV section was incubated in 100 µL of picrosirius red (Merck Pty Ltd, Kilsyth, Victoria, Australia) solution for 1 hour at room temperature to aid visualization of collagenous matrix. Sections were then briefly rinsed in 2 changes of acidified water (1% acetic acid), dehydrated in 2× 100% ethanol for 3 minutes each and 2× histolene for 2 minutes each, and coverslipped with DPX mounting media. Immunohistochemistry was performed on 4 µm sections, as previously described [21].

### Measurement of cardiomyocyte hypertrophy

The extent of cardiac myocyte hypertrophy, as measured by cross sectional area (CSA), was determined on haemotoxylin-eosin stained sections as previously published [21]. In brief, only myofibers with intact cellular membranes from field with circular capillary profiles and myofiber shapes were assessed and the circumferences of 20–30 cells per LV were traced and digitized to calculate mean CSA.

### Quantification of histological parameters

The accumulation of matrix (picrosirius red) and the extent of immunostaining of collagen I, collagen III, and 3-nitrotyrosine were quantified using computer-assisted image analysis software, as previously described [21]. Sections were scanned and digitized using Aperio ScanScope Console v.8.0.0.1058 (Aperio Technologies, Inc). Ten random non-overlapping fields from each section around the subendocardial region were captured using Aperio ImageScope v.8.0.39.1059 (Aperio Technologies, Inc) or Axioimager.A1 microscope attached to an AxioCam MRe5 digital camera (Carl Zeiss AxioVision, Germany) at ×230 magnification. Images were then exported and loaded onto a Pentium D Dell computer. An area of red on picrosirius red-stained (for matrix) or brown on immunostained sections (for collagen I and collagen III) were highlighted using a selective colour tool. Calculation of proportional area stained red or brown was determined using image analysis software AIS (Analytic Imaging Station version 6.0, Imaging Research Inc., Ontario, Canada) or AxioVs40LE (AxioVision version 4.5.0.0).

### NADPH oxidase activity

NADPH oxidase-dependent superoxide production in LV tissues was measured using lucigenin-enhanced chemiluminescence (LEC) as previously described [25]. Equal size of LV tissues were homogenized using glass homogenizer in the buffer containing 250 mM sucrose and 10 mM HEPES with protease inhibitors. Lysate was collected by centrifugation at 12,000 rpm for 10 mins at 4°C. Protein was quantitated and equal amount of lysate was transferred into a 96-well OptiPlate (Packard BioScience, Australia) with 200 µl Krebs-HEPES buffer in each well. 5 µM lucigenin and 100 µM NADPH were added into each well and the chemiluminescence was detected using a POLARstar OPTIMA plate reader (BMG Labtech, Offenburg, Germany). All the chemiluminescence data were normalised to protein concentration.

### Real-time quantitative polymerase chain reaction (PCR)

Real-time quantitative PCR was used to assess transcript levels of thioredoxin-interacting protein (TXNIP, NM_006472), Cu/Zn superoxide dismutase (SOD1, NM_017050), and glutathione peroxidase (Gpx1, NM_030826). A 20–25 µL of real-time PCR reaction included Brilliant SYBR Green QRT-PCR Master Mix as per manufacturer's instructions (Stratagene, USA). Real-time quantitations were performed using ABI Prism 7000 Sequence Detection System (Applied Biosystems, CA, USA) according to manufacturer's instructions. The fluorescence threshold value was calculated and the calculation of relative change in mRNA was performed using the delta-delta C_T_ method, with normalization for the housekeeping gene 18s. Nucleotide sequences of primers were as follows:

TXNIP (forward) 5′-AGGATTCTGTGAAGGTGATG-3′

TXNIP (reverse) 5′-TCTGACTGAGGACAGCTTCT-3′

SOD1 (forward) 5′-CGGTGCAGGGCGTCATTCACTT-3′

SOD1 (reverse) 5′-CCGCTGGACCGCCATGTTTCTT-3′

Gpx1 (forward) 5′-GGTGCTGGGCTCTGACTGCG-3′

Gpx1 (reverse) 5′-GCGCGCGGAGAAGGCATACA-3′

18S (forward) 5′-TCGAGGCCCTGTAATTGGAA-3′

18S (reverse) 5′-CCCTCCAATGGATCCTCGTT-3′

### ^33^P in situ hybridization

Synthesis of riboprobes and in situ hybridization were performed as previously described [25], [26]. Briefly, ^33^P-labelled antisense RNA probe for Txnip was generated by in vitro transcription (Promega, WI, USA) from linearized templates. Primers were designed using Oligo 6 primer design software (Molecular Biology Insight, CO, USA). Two rat Txnip probes were generated by RT-PCR, using rat kidney cDNA as template, to span the regions 1481–2004 (540 bp) and 2008–2384 (377 bp) of the rat Txnip sequence (NM_001008767). Purified riboprobe length was adjusted to approximately 150 bases by alkaline hydrolysis. *In situ* hybridization was performed on 4 µm thick sections of formaldehyde-fixed, paraffin-embedded LV tissue. Briefly, tissue sections were dewaxed in histolene, rehydrated in graded ethanol, and microwaved in 10 mM citrate buffer pH 6.0 on medium-high (600 to 700 W) for 5 min. Sections were washed in 0.1 M sodium phosphate buffer pH 7.2, fixed in 4% paraformaldehyde for 10 min, and washed again in phosphate buffer and milliQ water. After equilibration in P buffer (50 mM Tris-HCl pH 7.2 and 5 mM EDTA pH 8.0), slides were incubated with 125 µg/ml Pronase E (Sigma) in P buffer pH 7.2, refixed in 4% paraformaldehyde for 10 min, rinsed in milliQ water, dehydrated in 70% ethanol, and air dried. Hybridization of the riboprobe to the pretreated tissue was performed overnight at 60°C in 50% formamide-humidified chambers. Sense probes were used on an additional set of tissue sections as controls for nonspecific binding. After hybridization, slides were washed, incubated with RNase A, dehydrated in graded ethanol, air dried, and exposed to Kodak Biomax MR autoradiographic film (Kodak, Rochester, NY) for 3 days.

### Quantitative autoradiography

Densitometry of autoradiographic images obtained by *in situ* hybridization was performed by computer-assisted image analysis using Micro Computing Imaging Device (MCID; Imaging Research, Ontario, Canada) as previously described [25]. In brief, in situ autoradiographic images were placed on a uniformly illuminating fluorescent light box (Northern Light Precision Luminator model C60) and captured using a video camera (Dage MTI CCD72) connected to an IBM AT computer with a 512×512 pixel array imaging board with 256 grey levels. After calibration by construction of a curve of optical density versus radioactivity density using Amersham ^14^C microscale autoradiography standard, which were co-exposed with the hybridized sections, quantification of digitalized autoradiographic images was performed with the MCID software and expressed as nCi/g.

### Western blot

Western blots were performed as previously described [27]. Protein concentration of heart tissue homogenates were determined using Bio-Rad Bradford Protein Assay (Bio-Rad, CA, USA). Samples with equal concentration of protein were subjected to SDS-PAGE and western blot analysis with rabbit polyclonal Txnip antibody overnight at 4°C (1∶1000: Invitrogen, CA, USA). Following incubation with anti-rabbit secondary antibody (1∶2500: Dako, Golstrup, Denmark) for 1 hour at room temperature, proteins were detected by ECL detection system. The membranes were reprobed with pan-actin (1∶500: Neomarkers, CA, USA), which served as loading control. The bands corresponding to Txnip (50 kDa) and pan-actin (42 kDa) were quantitated by densitometry using Quantity One Software (Bio-Rad, CA, USA) and expressed as the ratio of the loading control. At least six samples were analysed from each group in four separate gels.

### Statistical analyses

Data were expressed as mean ± standard error of mean (SE) unless otherwise stated. Differences between groups were determined by one-way analysis of variance (ANOVA) with Fisher PLSD *post hoc* comparison using Statview II + Graphics package (Abacus Concepts, Berkeley, CA). A value of *P*<0.05 was considered as statistically significant.

## Results

### Animal characteristics of homozygous Ren-2 rats with or without diabetes for 6 weeks

All rats were hypertensive with elevated systolic blood pressure. Blood glucose was elevated to a similar extent in diabetic animals. Body weight and heart weight, indexed to body weight (HW∶BW) were reduced in diabetic rats. DiOHF treatment did not significantly alter BGL, SBP, BW or HW∶BW in either control or diabetic animals (Table 1).

**Table 1:** Animal characteristics of control and diabetic rats treated with vehicle or DiOHF.

	Control	Control + DiOHF	Diabetic	Diabetic + DiOHF
***N***	12	7	10	11
**BGL (mmol/L)**			32.8 ± 0.1	31.2 ± 0.6
**SBP (mmHg)**	245 ± 6.2	236.6 ± 12.2	235.8 ± 20.3	236.7 ± 19.6
**BW (g)**	318.00 ± 12.12	301.14 ± 13.35	224.67 ± 8.13*	217.82 ± 7.01*
**HW∶BW**	0.52 ± 0.014	0.53 ± 0.061	0.41 ± 0.017*	0.41 ± 0.008*
**Lung∶BW**	0.51 ± 0.025	0.49 ± 0.022	0.58 ± 0.033	0.61 ± 0.033

Values are Mean ± SE; BGL, Blood glucose level; SBP, Systolic blood pressure; BW, Body weight, HW, Heart weight.

*P<0.05 vs control (non-diabetic) rats.

### DiOHF attenuated left ventricular diastolic dysfunction in diabetic Ren-2 rats as assessed by cardiac catheterization and echocardiography

Chamber compliance, a measure of diastolic function was significantly reduced in diabetic rats (*P*<0.05) when compared to control rats (Table 2b, Fig. 1). Chamber compliance is inversely proportional to the slope of end-diastolic pressure volume relationship (EDPVR). Treatment of diabetic rats with DiOHF improved chamber compliance to levels comparable to control rats (*P*<0.05; Table 2b, Fig. 1). Active relaxation, as measured by Tau τ, was significantly prolonged in diabetic compared to control rats. DiOHF treatment significantly attenuated the increase in Tau τ in diabetic animals (*P*<0.05; Table 2b).

**Figure 1:** Representative pressure volume (PV) loops during preload reduction. Note the steeper slope of EDPVR (green line) and rightward shift in the diabetic group (C) compared to control (A). An increase in the slope of EDPVR indicated decreased chamber compliance as seen in the diabetic animals which was reduced with DiOHF treatment (D). *P<0.05 vs control (non-diabetic) rats; †*P*<0.05 vs diabetic rats.

**Table 2:** Steady state and load insensitive parameters of cardiac contraction and relaxation.

	Control	Control + DiOHF	Diabetic	Diabetic + DiOHF
**A**				
***N***	9	5	8	10
**HR (bpm)**	295 ± 15	278 ± 30	246 ± 12*	245 ± 8
**EDV (µL)**	207.42 ± 16.98	203.94 ± 30.35	260.38 ± 31.99	225.68 ± 18.63
**EDP (mmHg)**	4.62 ± 0.51	5.20 ± 0.55	10.05 ± 0.91*	5.94 ± 0.57†
**B**				
**dP/dt max (mmHg / sec)**	5394 ± 827	4115 ± 632	5199 ± 872	5207 ±337
**Tau τ (msec) Weiss**	14.2 ± 0.8	14.5 ± 1.0	17.0 ± 0.8*	14.7 ± 0.6†
**EDPVR (slope-mmHg/µL)**	0.026 ± 0.004	0.030 ± 0.005	0.060 ± 0.011*	0.027 ± 0.002†
**PRSW (slope-mmHg)**	106 ± 15	123 ± 28	44 ± 7*	71 ± 8

Values are Mean ± SE; A: HR, Heart rate; EDV, End-diastolic volume; EDP, End-diastolic pressure; B: dP/dt max, the maximal rate of pressure change; Tau, time constant of pressure decay; PRSW, slope of preload recruitable stroke work relationship; EDPVR, slope of end-diastolic pressure volume relationship.

*P<0.05 vs control (non-diabetic) rats;

† *P*<0.05 vs diabetic rats.

Diastolic function, assessed using Doppler echocardiographic examination, showed a significant reduction in E to A ratio in diabetic animals when compared to control rats (*P*<0.05) with a trend to improvement following DiOHF treatment (Table 3, Fig. 2). Diabetic rats demonstrated impaired relaxation with prolonged deceleration time (DT) of early (E) diastolic filling compared to control rats (*P*<0.05), which was significantly improved with DiOHF treatment (*P*<0.05; Table 3). There were no significant differences in any cardiac parameters measured in control rats when compared to control rats treated with DiOHF.

**Figure 2:** Representative apical view pulsed wave Doppler studies. In control rats (A) “normal” left ventricular (LV) filling pattern were observed, whereas diabetic rats (B) had reduced LV function. These changes were distinguished by delayed ventricular relaxation, characterized by reduction in the E wave and an increase in the late atrial A wave and prolongation of the deceleration time. Treatment with DiOHF showed improvement in LV function of diabetic rats (C).

**Table 3:** Echocardiographic parameters in control and diabetic rats, treated with or without DiOHF for 6 weeks.

	Control	Control + DiOHF	Diabetic	Diabetic + DiOHF
**FAC (%)**	66.99 ± 2.30	71.62 ± 3.90	71.07 ± 2.78	74.42 ± 3.26
**LVID d**	0.58 ± 0.02	0.56 ± 0.03	0.64 ± 0.02*	0.58 ± 0.02
**LVID s**	0.27 ± 0.01	0.22 ± 0.02	0.26 ± 0.02	0.20 ± 0.02†
**FS % (M mode)**	53.38 ± 1.75	61.57 ± 3.08	59.89 ± 2.63	66.00 ± 2.98
**EF (%)**	80.46 ± 1.41	79.06 ± 2.68	75.79 ± 0.71	81.69 ± 1.42
**Dec T (ms)**	36.75 ± 3.90	37.33 ± 4.63	45.29 ± 2.06*	31.83 ± 1.19†
**E/A ratio**	1.85 ± 0.29	1.53 ± 0.03	1.41 ± 0.08*	1.72 ± 0.12

Values are Mean ± SE; FAC, Fractional Area Change; LVID d, Left Ventricular Internal end Diastolic dimension; LVID s, Left Ventricular Internal end Systolic dimension; EF, Ejection Fraction; FS, Fractional Shortening; Dec T, Deceleration time.

*P<0.05 vs control (non-diabetic) rats;

† *P*<0.05 vs diabetic rats.

Heart rate was significantly reduced in diabetic rats when compared to control rats (*P*<0.05). DiOHF treatment did not significantly alter heart rate in either diabetic or control animals (Table 2a). End-diastolic pressure (EDP) was significantly elevated in diabetic compared to control rats (*P*<0.05) and was attenuated by DiOHF in diabetic rats.

### DiOHF ameliorated myocardial fibrosis and cellular hypertrophy in diabetic Ren-2 rats

Diabetes was associated with a significant increase in myocardial fibrosis as evidenced by greater proportional area of interstitial collagen I and III immunostaining (Fig. 3 and 4) and extracellular matrix deposition (data not shown). Diabetic rats also displayed cellular hypertrophy with increased cardiomyocyte cross-sectional area when compared with control rats (*P*<0.05; Fig. 5). DiOHF treatment significantly attenuated myocardial fibrosis and cellular hypertrophy (*P*<0.05 versus diabetic).

**Figure 3:** Immumohistochemistry staining for collagen type I. (A) Representative images. Brown region represents positive immunostaining for collagen type I which was substantially increased in diabetic rats and reduced by DiOHF treatment. The amount of collagen type I was found to be similar in control and control-treated rats. Collagen type I interstitial accumulation as assessed by percentage proportional area showing positive immunostaining in control and diabetic rats treated with or without DiOHF (B). Data expressed as mean ± SE. *P<0.05 vs control (non-diabetic) rats; †*P*<0.05 vs diabetic rats. Original magnification ×200.

**Figure 4:** Immunohistochemistry staining for collagen type III. (A) Representative images. Brown region represents positive immunostaining for collagen type III which was substantially increased in diabetic rats and reduced by DiOHF treatment. The amount of collagen type III was found to be similar in control and control-treated rats. Collagen type III interstitial accumulation as assessed by proportional area on sections showing positive immunostaining in control and diabetic rats treated with or without DiOHF (B). Data expressed as mean ± SE. Data expressed as mean ± SE. *P<0.05 vs control (non-diabetic) rats; †*P*<0.05 vs diabetic rats. Original magnification ×200.

**Figure 5:** Representative images for myocyte hypertrophy. (A) Diabetic rats demonstrated myocyte hypertrophy as evidenced by increased cross sectional area when compared with control rats. Treatment with DiOHF reduced cross sectional area in diabetic rats but had no effect on control rats. (B) Quantitative data for myocyte cross sectional area. *P<0.05 vs control (non-diabetic) rats; †*P*<0.05 vs diabetic rats. Original magnification ×200.

### DiOHF attenuated cardiac oxidative stress in diabetic Ren-2 rats, independent of changes in the gene expression of intracellular antioxidant enzymes

The presence of diabetes resulted in significant induction of intracellular oxidative stress as measured by increased tissue localisation of 3-nitrotyrosine and NADPH oxidase-dependent superoxide production (*P*<0.05 versus control), which were significantly attenuated by DiOHF in diabetic rats (*P*<0.05; Fig. 6). Similarly, Txnip mRNA and protein expression levels were significantly increased in diabetic compared to control rats (*P*<0.05 versus control) and were attenuated by DiOHF treatment (Fig. 8 and 9). No significant differences were observed in the control rats when compared to control-treated rats.

**Figure 6:** Measurements of oxidative stress. Representative images for the localization of 3-nitrotyrosine in LV tissues, as assessed by the proportional area of positive immunostaining in control and diabetic rats treated with or without DiOHF (A). The marked increase in positive immunostaining (brown region) for 3-nitrotyrosine in diabetic rats was reduced by DiOHF treatment. The amount of 3-nitrotyrosine was found to be comparable in control and control-treated Ren-2 rats (B). Original magnification ×200. (C) NADPH-activated superoxide production in LV tissues as measured by lucigenin-enhanced chemiluminescence. Data expressed as mean ± SE. *P<0.05 vs control (non-diabetic) rats; †*P*<0.05 vs diabetic rats.

Diabetic animals demonstrated a marked increase in the gene expression of intracellular antioxidant enzymes such as superoxide dismutase (SOD1) and glutathione peroxidase (Gpx1) when compared to control rats (Fig. 7). SOD1 and Gpx1 mRNA levels were not changed by DIOHF treatment in diabetic rats.

**Figure 7:** Intracellular antioxidants mRNA gene expression. (A) Measurement of Cu/Zn-superoxide dismutase (SOD1) and (B) gluthathione peroxidase (Gpx1) mRNA by real time RT-PCR, normalized to the housekeeping gene 18s. Diabetic rats demonstrated increased gene expression of SOD1 and Gpx1, which were not affected by DiOHF. Data expressed as mean ± SE. *P<0.001 vs control (non-diabetic) rats.

**Figure 8:** Txnip mRNA gene expression. (A) Representative autoradiographs from *in situ* hybridization of Txnip. The magnitude of gene expression is indicated quantitatively as a pseudocolourized computer image (blue, nil; green, low; yellow, moderate; red, high). (B) Quantitation of Txnip gene expression by quantitative autoradiography. (C) Measurement of Txnip mRNA by real time RT-PCR, normalized to the housekeeping gene 18s. Data expressed as mean ± SE. *P<0.05 vs control (non-diabetic) rats; †*P*<0.05 vs diabetic rats.

**Figure 9:** Txnip protein expression. (A) Representative western blot and (B) quantitation of Txnip normalized to loading control pan-actin. The significant increase in Txnip protein in diabetic rats was moderately reduced by DiOHF treatment. Data expressed as mean ± SE. *P<0.05 vs control (non-diabetic) rats.

## Discussion

Clinically, DCM is characterized by early abnormalities in LV diastolic function that ultimately lead to chronic heart failure with subtle or no changes in LV systolic function [28]. The most prominent cardiac remodelling event associated with these functional alterations is myocardial fibrosis with the accumulation of extracellular matrix components including collagen types I and III [28], [29]. The present study demonstrates that suppression of oxidative stress with DiOHF, a broad spectrum antioxidant, in an experimental model of diastolic heart failure due to diabetes, led to improved chamber compliance, reduced myocyte hypertrophy and collagen deposition. To our knowledge, this is the first study showing that oral antioxidant therapy with DiOHF prevents hyperglycemia-induced oxidative stress-mediated myocardial injury and may represent a novel therapy to explore clinically.

The pathogenesis of LV dysfunction in diabetic hearts has not been fully elucidated. The correlation between hyperglycemia and oxidative stress demonstrated in clinical and experimental studies may be due to the upregulation of local renin-angiotensin systems (RAS) [30]. Here, we have demonstrated that DiOHF treatment did not significantly alter cardiac function and structure in non-diabetic Ren-2 rats in the presence of an enhanced local RAS alone. However, induction of diabetes in Ren-2 rats resulted in marked deterioration of cardiac pathology, which was significantly attenuated by DiOHF treatment. The sensitization of local RAS by hyperglycemia has been associated with upregulation of the AT_1_ receptor and increase in ROS via stimulation of NADPH oxidase activity [30], [31]. In the present study, localization of 3-nitrotyrosine, a biomarker of oxidative stress was markedly reduced in the myocardium of diabetic Ren-2 rats treated with DiOHF, in conjunction with a reduction in interstitial collagenous matrix deposition. We also demonstrated that DiOHF led to a reduction in NADPH oxidase-dependent superoxide production in the LV sections from diabetic Ren-2 rats. These results are in accord with Wang and colleagues [20], who established that the antioxidant actions of DiOHF were responsible for the attenuation of myocardial ischemia-reperfusion injury.

The exact mechanisms leading to the observed structural and functional improvements in DCM with DiOHF therapy remain speculative. Flavonols have long been recognized for their ability to scavenge superoxide radicals and to inhibit enzymes responsible for the production of oxygen radicals [32], [33]. DiOHF may exert pleiotropic effects in the diabetic Ren-2 hearts not only through increasing ROS scavenging or decreasing NADPH oxidase-dependent superoxide production but also perhaps by restoring the function of intracellular enzymatic or non-enzymatic antioxidants. The thioredoxin system, one of the major intracellular antioxidant defense mechanisms, prevents oxidative stress by removing oxygen radical intermediates. However, the antioxidative function of thioredoxin is inhibited when thioredoxin interacting protein (Txnip) binds to the catalytic site of the reduced form of thioredoxin [34], [35]. Txnip has been shown to be increased in the hearts of streptozotocin-induced diabetic mice, suggesting that diabetes-induced alterations in redox balance may contribute to the pathological processes in DCM [36]. Consistent with previous findings in diabetic Ren-2 kidneys, Txnip mRNA and protein expression levels were elevated in the hearts of diabetic Ren-2 animals [26], [37]. We further demonstrated that Txnip overexpression in the diabetic Ren-2 hearts was prevented when treated with DiOHF, possibly leading to the restoration of thioredoxin activity [26]. In addition, the enhanced gene expression of Cu/Zn-superoxide dismutase and glutathione peroxidase in the presence of diabetes suggests that there could be compensatory mechanisms to protect against oxidative stress [38], [39]. The expression of these antioxidant enzymes remained higher in diabetic-treated than in control-untreated Ren-2 animals, despite notable restoration of cardiac redox balance. Although we were unable to evaluate the functional integrity of these antioxidant enzymes, we cannot exclude the possibility that these enzymes may have reduced or impaired function as a result of post-translational modifications, such as glycation, and nitration, by different reactive intermediates commonly present in the diabetic milieu [40], [41], [42], [43].

Current therapies available for the prevention of CHF in diabetic patients target glycemic and blood pressure control, predominantly through blockade of the RAS [3], [44]. For instance, chronic AT_1_ receptor blockade by candesartan in type 2 diabetic patients reduced myocardial fibrosis correlated with improved diastolic function [45]. However, large-scale clinical trials, such as I-PRESERVE (Irbesartan in HF with Preserved Systolic Function) and CHARM-Preserved (Candesartan in Heart Failure to Affect Reduction in Morbidity and Mortality), showed moderate or no improvement in cardiovascular mortality and morbidity among patients with heart failure and preserved LV ejection fraction (HF-PEF) [46], [47]. Retrospective cohort studies from these clinical trials demonstrated that diabetes was present in approximately 28% of HF-PEF patients and was identified as an independent predictor of cardiovascular mortality and HF hospitalization [48], [49]. These treatments are to a certain extent effective at delaying the onset of CHF in patients presented with systolic dysfunction (LVEF<40%) but not much is known about the impact of these therapies on the various stages of diastolic dysfunction. This further highlights the absence of therapeutic interventions for diastolic heart failure among diabetic patients [50]. Here, diabetic Ren-2 rats that were administered a therapeutic dose of DiOHF demonstrated up to 55% improvement in chamber compliance when compared to untreated diabetic Ren-2 rats. The passive diastolic properties of the LV were normalized to the level observed in control Ren-2 group. However, whether DiOHF antioxidant might provide additional therapeutic benefits when added to angiotensin-converting enzyme inhibition or angiotensin receptor blockade have yet to be assessed.

Echocardiography and invasive pressure-volume (PV) loops analysis were performed to investigate the active and passive properties of the LV during diastole, along with assessment of systolic performance. During early diastolic dysfunction, impaired LV relaxation and compliance is denoted by reduced magnitude of E wave, compensated by increased atrial contraction, resulting in reduced E∶A ratio, as observed in diabetic Ren-2 animals [28], [51]. Also, impaired relaxation with prolonged deceleration time (DT) was observed in diabetic Ren-2 animals. However, interpretation of intrinsic diastolic properties using echocardiography is limited due to the preload dependence [28], [52] and recently highlighted heart rate dependence [53] of the Doppler LV filling parameters. Consequently, load-insensitive measurements of chamber compliance were determined by examining end-diastolic pressure-volume relationship (EDPVR) over varying loading conditions [54]. We demonstrated that the marked reduction in chamber compliance in Ren-2 diabetic animals was attenuated by treatment with DiOHF antioxidant at the time point assessed. The rate of relaxation, measured by time constant of relaxation (Tau) during the active phase of diastole, was also prolonged in Ren-2 diabetic animals.

These data are consistent with the manifestation of LV diastolic dysfunction frequently found in diabetic patients without other known cardiac defects, such as atherosclerosis or hypertension [28], [55]. Martos *et al.* [56] demonstrated that markers of collagen turnover associated with active fibrotic processes were elevated in patients diagnosed with more severe phases of diastolic dysfunction. Using non-invasive monitoring of myocardial fibrosis in diabetic patients, the change in LV chamber compliance has been correlated to regulation of collagen turnover [57]. In our study, the diabetic Ren-2 rats treated with DiOHF demonstrated significant reduction in cardiac myocyte hypertrophy and collagen types I and III. These structural effects may have contributed to the observed improvement in chamber compliance.

In contrast, load-dependent indices of systolic function examined by fractional shortening (FS) and fractional area change (FAC) showed no significant differences among diabetic and control Ren-2 animals. Similarly, the LV ejection fraction (EF) was within the normal range (EF>60%) across all groups. The assessment of systolic function by conventional echocardiography is not only influenced by cardiac contractility but other factors including loading conditions and heart rate [58]. In the present study, the ‘gold standard’ invasive PV loops analysis of diabetic Ren-2 rats showed a reduction in the slope of preload recruitable stroke work relationship (PRSW), indicative of subtle differences in cardiac contractility, that were not detected by echocardiography. Further, DiOHF treatment tended to improve PRSW in diabetic rats indicating improved systolic function. These findings are consistent with clinical findings where diastolic dysfunction is often accompanied by systolic dysfunction in diabetes.

The current study has established the potential clinical utility of antioxidant therapy in preventing the development of diabetic cardiomyopathy, despite persistent hypertension and hyperglycemia. The early induction of therapy following onset of diabetes may account for the vast improvement in functional parameters measured in diabetic-treated Ren-2 animals. However, it remains to be explored if the current therapy would continue to preserve cardiac function in the presence of sustained severe hyperglycemia among diabetic subjects. Hence, it would be of considerable interest to examine the effect of DiOHF therapy on the myocardium in the presence of diabetes at a later time point.

In conclusion, diabetic Ren-2 rats treated with DiOHF demonstrated improved diastolic function with a trend towards improved systolic function. DiOHF therapy reduced the accumulation of extracellular matrix components, particularly collagen types I and III, which are associated with myocardial fibrosis observed in diabetic Ren-2 rats. These findings suggest that DiOHF therapy is cardioprotective in diabetic Ren-2 rats, and these data may have implications in the clinical setting with clinical trials using similar antioxidants in the context of diastolic heart failure has just begun (GRAPEVINE-HF, NCT01185067).
